This article has been retracted.

# Clinical and Dermoscopic Evaluation of Periorbital Melanosis and Its Psychological Impact and Effect on Quality of Life: A Descriptive Study

**DOI:** 10.7759/cureus.74625

**Published:** 2024-11-27

**Authors:** Saumya Banchhor, Sanjeev Gupta, Aneet Mahendra

**Affiliations:** 1 Dermatology, Maharishi Markandeshwar Institute of Medical Sciences and Research, Mullana, IND

**Keywords:** body dysmorphic disorder, dermoscopy, perceived stress scale (pss), periorbital melanosis, wood's lamp

## Abstract

Introduction: Periorbital melanosis (POM) is a poorly defined condition that is becoming an increasing aesthetic concern. With its multifactorial origin, it necessitates a thorough assessment of targeted multimodal treatments. The psychological impact and underlying pathogenesis have been underexplored, as evidenced by the gap between the roughly 100 indexed articles and the 150 million search engine results on treatments for dark circles. This descriptive study aims to explore the clinical and dermoscopic evaluation of POM and its impact on quality of life.

Methods: This descriptive prospective, tertiary hospital-based study included 250 patients with POM attending the Dermatology Outpatient Department. After obtaining informed consent, patients were subjected to clinical assessment, hematological investigations, and Wood's lamp (by Dermaindia, Chennai, India) examination. The dermatoscopic examination was done using a Dino-Lite video dermatoscope AF4515ZT+WF-20 (AnMo Electronics Corporation, Taipei, Taiwan). Quality of life was measured using the Melasma Quality of Life (MELASQoL) scale, and the psychological impact was assessed using the Perceived Stress Scale (PSS) and Body Dysmorphic Disorder Questionnaire-Dermatology Version (BDDQ-DV).

Results: Among 250 patients, 179 (71.6%) were female and 71 (28.4%) were male, with a mean age of 30.53±9.29 years and a disease duration of 6.82±5.04 years. Constitutional POM was the most common type observed in 219 (87.6%) patients. Dermoscopy showed blotches in 166 (66.4%), telangiectasia in 211 (84.4%), and exaggerated skin markings in 17 (6.8%), and no atrophic changes were observed. Mean MELASQoL and PSS scores were 25.63±10.52 and 16.64±3.27, respectively; four (1.6%) patients had body dysmorphic disorder.

Conclusion: POM has a complex etiology with multiple underlying mechanisms. Thorough clinical assessment enables accurate diagnosis and a targeted treatment approach. Thus, unnecessary medications and procedures can be avoided by first understanding the underlying pathophysiology. Further studies are warranted in the Indian population with POM, as the skin type, demography, and socioeconomic status are diverse. Various proposed classifications are available but do not cater to the Indian skin type; hence, further research is due.

## Introduction

Periorbital melanosis (POM) is an ill-defined entity that presents as bilateral round or semicircular homogenous brown or dark brown pigmented macules involving the periorbital area and sometimes including the malar area, temporals, and lateral nasal root [1]. POM has many synonyms which include periorbital hypermelanosis, periocular hyperpigmentation, periorbital darkening, under-eye dark circles, or idiopathic cutaneous hyperchromia of the orbital region (ICHOR).

In the past few years, aesthetic facial concerns have accounted for the majority of dermatological consultations, among which the uprising concern is the one that is called "dark circles under the eyes" or POM. Women are more frequently affected by POM than men and more likely to seek medical advice. The prevalence of Indian women with a moderate to severe grade of POM is as high as 50%.

POM can either have exogenous or endogenous aetiologies. Some of the contributing factors include genetic predisposition, lifestyle influence, sun exposure, ocular hypotensive drugs, systemic illness, and post-inflammatory melanosis following atopic dermatitis or allergic contact dermatitis. Increase in periorbital vasculature and pigmentation, shadow effect due to the laxness of the skin, prolapse of periocular adipose tissue, and tear trough formation with aging all contribute to POM development [2].

## Materials and methods

Study design

This was a descriptive prospective study conducted at the Dermatology Outpatient Department of Maharishi Markandeshwar Institute of Medical Sciences and Research, Mullana, Ambala, Haryana, India, over one year and seven months from January 2023 to July 2024.

Inclusion criteria

This study included cases of POM of either sex with ages ranging from 18 to 60 years. Patients with a disease duration of more than one year were included in the study.

Exclusion criteria

Patients either under 18 years or over 60 years of age were excluded from the study. Pregnant or lactating women, patients with other additional eyelid dermatoses, and patients with other hyperpigmentary dermatoses of the face were also excluded from the study.

Participants were thoroughly explained the study objectives, and proper consents were obtained. With due permission from the Institutional Ethical Committee of Maharishi Markandeshwar Institute of Medical Sciences and Research (approval number: 2547), 250 clinically diagnosed patients of POM were included.

Study tool and data collection

A detailed proforma was used to gather the patient's medical history, including family history, associated systemic illnesses, treatment history, and lifestyle influences associated with POM. Clinical examination was done to assess the anatomical structure, type of POM, site of involvement, color of pigmentation, and severity of hyperpigmentation. The assessment was conducted using a Wood's lamp (by Dermaindia, Chennai, India) and by performing a manual eyelid stretch test. Hematological investigation included hemoglobin and thyroid-stimulating hormone (TSH). The dermatoscopic examination was done using a Dino-Lite video dermatoscope AF4515ZT+WF-20 (AnMo Electronics Corporation, Taipei, Taiwan). Quality of life was measured using the Melasma Quality of Life (MELASQoL) scale, and the psychological impact was assessed using the Perceived Stress Scale (PSS) and Body Dysmorphic Disorder Questionnaire-Dermatology Version (BDDQ-DV).

Statistical analysis

The data was analyzed using IBM SPSS Statistics for Windows, Version 28.0 (Released 2021; IBM Corp., Armonk, New York, United States) and Excel, Version 2019 (Microsoft Corporation, Redmond, Washington, United States). Descriptive statistical methods were used to encapsulate the data, the continuous variables were presented using the median, mean, and standard deviation, and the categorical variables were expressed in frequency and proportion. The chi-squared (χ2) results were obtained using the chi-squared test which was used to analyze categorical variables, and the F-value was derived using the one-way ANOVA to analyze continuous variables.

## Results

Sociodemography

Among the 250 patients aged 18-60 years, the majority were between 25 and 45 years (138, 55.2%), with a mean of 30.53±9.29 years. The mean duration of the disease was 6.82±5.04 years with a majority of 107 (42.8%) patients having a duration of less than five years (Table 1).

**Table 1:** Distribution of patients with periorbital melanosis in terms of sociodemographic details

Variables	Frequency, n (%)
Age (years)	
18-25	87 (34.8%)
25-45	138 (55.2%)
45-60	25 (10%)
Gender	
Female	179 (71.6%)
Male	71 (28.4%)
Area of living	
Rural	150 (60%)
Urban	100 (40%)
Occupation	
Homemaker	91 (36.4%)
Skilled professionals	47 (18.8%)
Unskilled professionals	14 (5.6%)
Student	98 (39.2%)
Family history	
Absent	146 (58.4%)
Present	104 (41.6%)
Familial consanguinity	
Absent	246 (98.4%)
Present	4 (1.6%)

Aetiological factors

The impact on POM by aggravating factors, lifestyle influences, and the treatments used in the past were noted (Table 2). In terms of concomitant diseases associated with POM, 26 (10.4%) were anemic, 24 (9.6%) gave a history of acute illness before the formation of POM (dengue and chikungunya), 22 (8.8%) had thyroid disorders, and eight (3.2%) had atopic diathesis. Elevated serum TSH was observed in two (0.8%) and decreased serum TSH in five (2%).

**Table 2:** Distribution of patients with periorbital melanosis based on aggravating factors, lifestyle influences, and treatments used in the past

Variables	Frequency, n (%)
Effect of menstruation	
Absent	108 (60.3%)
Present	71 (39.6%)
Drug history	
Absent	202 (80.8%)
Present	48 (19.2%)
Sun exposure	
Absent	178 (71.2%)
Present	72 (28.8%)
Sleep hours	
<6 hours	64 (25.6%)
≥6 hours	186 (74.4%)
Screen time	
<8 hours	154 (61.6%)
≥8 hours	96 (38.4%)
Spectacle use	
Absent	169 (67.6%)
Present	81 (32.4%)
Frequent eye rubbing	
Absent	151 (60.4%)
Present	99 (39.6%)
Self-used topical medication	
Absent	156 (62.4%)
Present	94 (37.6%)
Home remedies	
Absent	125 (50%)
Present	125 (50%)
Cosmetic use	
Absent	165 (66%)
Present	85 (34%)

Clinical and dermoscopic observation

The physical assessment of POM includes the site of involvement, the color of pigmentation, the physical changes, and the grade of POM (Figure 1, Table 3). Wood's lamp examination observed 180 (72%) patients with the dermal type and 70 (28%) with the epidermal type of pigmentation in POM (Figure 2 and Figure 3). The dermoscopy examination of POM includes the pattern of pigmentation (Figure 4 and Figure 5), the vasculature, and the skin surface changes (Table 4).

**Figure 1:** Mild grade of periorbital melanosis

**Table 3:** Distribution of variables in the physical assessment of periorbital melanosis

Variable	Frequency, n (%)
Site of involvement	
Both eyelid	11 (4.4%)
Both eyelids, lateral nasal root	130 (52%)
Lateral nasal root	34 (13.6%)
Lower eyelid, lateral nasal root	58 (23.2%)
Upper eyelid, lateral nasal root	17 (6.8%)
Color of pigmentation	
Bluish grey	4 (1.6%)
Brown	174 (69.6%)
Brown, brownish black	38 (15.2%)
Brownish black	34 (13.6%)
Violaceous	0 (0%)
Physical changes	
Shadow	15 (6%)
Shadow, visible lower eyelid bulging	1 (0.4%)
Tear trough	154 (61.6%)
Tear trough, dermatochalasis	1 (0.4%)
Tear trough, shadow	63 (25.2%)
Tear trough, visible lower eyelid bulging	11 (4.4%)
Visible lower eyelid bulging	5 (2%)
Type of periorbital melanosis	
Constitutional	219 (87.6%)
Post-inflammatory	22 (8.8%)
Shadow	7 (2.8%)
Vascular	2 (0.8%)
Grade of periorbital melanosis	
Mild	144 (57.6%)
Moderate	95 (38%)
Severe	11 (4.4%)
Very severe	0 (0%)

**Figure 2:** Tear trough type of periorbital melanosis

**Figure 3:** Tear trough pigmentation getting accentuated on Wood's lamp examination

**Figure 4:** Telangiectasia (white arrow) and coarse speckled pigmentation (within while circle) seen on dermoscopy

**Figure 5:** Exaggerated pigment network pattern seen on dermoscopy (white arrow)

**Table 4:** Distribution of dermoscopic examination in periorbital melanosis

Variable	Frequency, n (%)
Pattern of pigmentation	
Blotches	166 (66.4%)
Coarse speckled	14 (5.6%)
Exaggerated pigment network	27 (10.8%)
Fine speckled	30 (12%)
Globules	13 (5.2%)
Vasculature	
Superficial dilated veins	11 (4.4%)
Telangiectasia	183 (73.2%)
Telangiectasia, superficial dilated veins	28 (11.2%)
Absent	28 (11.2%)
Skin surface changes	
Exaggerated skin marking	17 (6.8%)
Absent	233 (93.2%)

Quality of life and psychological impact

The MELASQoL, PSS, and BDDQ-DV scoring were used to assess the quality of life and the psychological impact in patients with POM (Table 5). A significant association was found between the severity of POM and the MELASQoL score (p=0.00; χ2=48.522); however, no significant association was observed between the POM severity and PSS score (p=0.57; χ2=4.790) (Table 6). In addition to this, a significant association was found between screen time and the severity of POM (p=0.004; F=5.562) (Table 7).

**Table 5:** Distribution of psychological impact and quality of life among patients with periorbital melanosis MELASQoL: Melasma Quality of Life; PSS: Perceived Stress Scale; BDDQ-DV: Body Dysmorphic Disorder Questionnaire-Dermatology Version

Variable	Frequency, n (%)	Mean±standard deviation
MELASQoL score		
Mild impairment (10-39)	229 (91.6%)	25.6320±10.52481
Moderate impairment (40-55)	18 (7.2%)	
Severe impairment (56-70)	3 (1.2%)	
PSS score		
Much lower than average (0-7)	0 (0%)	16.6440±3.27784
Slightly lower than average (8-11)	14 (5.6%)	
Average (12-15)	92 (36.8%)	
Slightly higher than average (16-20)	114 (45.6%)	
Much higher than average (21 and over)	30 (12%)	
BDDQ-DV score		
No	246 (98.4%)	-
Yes	4 (1.6%)	

**Table 6:** Association of MELASQoL and PSS scoring with the severity of periorbital melanosis MELASQoL: Melasma Quality of Life; PSS: Perceived Stress Scale

Variable	Frequency, n (%)			P-value
	Mild (grade 1)	Moderate (grade 2)	Severe (grade 3)	
MELASQoL score				
Mild impairment	141 (56.4%)	83 (33.2%)	5 (2%)	0.00
Moderate impairment	0 (0%)	13 (5.2%)	5 (2%)	
Severe impairment	2 (0.8%)	0 (0%)	1 (0.4%)	
PSS score				
Much lower than average	0 (0%)	0 (0%)	0 (0%)	0.57
Slightly lower than average	6 (2.4%)	8 (3.2%)	0 (0%)	
Average	51 (20.4%)	38 (15.2%)	3 (1.2%)	
Slightly higher than average	69 (27.6%)	38 (15.2%)	7 (2.8%)	
Much higher than average	17 (6.8%)	12 (4.8%)	1 (0.4%)	

**Table 7:** Association of screen time with the severity of periorbital melanosis

Severity of periorbital melanosis	Screen time (hours), mean±standard deviation	P-value
Mild (grade 1)	3.09±2.07	0.004
Moderate (grade 2)	5.32±5.27	
Severe (grade 3)	6.62±3.37	

Owing to the aesthetic concerns, 108 (43.2%) patients were willing to invest in various POM treatments.

## Discussion

The cutaneous and structural changes of the periorbital region have a crucial role in perceiving the age of an individual. Darkening of the infraorbital skin can create a fatigued and less youthful appearance, making it an increasing aesthetic concern for many.

A gender imbalance was observed with 179 (71.6%) women affected by POM suggesting a higher prevalence among women or a greater concern in women than men. POM is common in the 16-30-year age group, owing to the physiological changes occurring during puberty and pregnancy [1]. However, driven by various aging concerns, it peaks again in the 45-60-year age range. POM is a significant cosmetic concern for young adults, especially for those preparing for marriage. As a chronic condition, it may persist for years if the underlying cause is not addressed. It is not solely an urban cosmetic concern; rising cases are seen in rural areas as well. Since the study location was based in a rural area, 150 (60%) patients were residents of the same. Additionally, with the increasing availability of online digital platforms in rural regions, they too have access to browse the current trends which can cater to their aesthetic concerns.

A study delineated the autosomal dominant trait of POM, wherein they found 22 members with POM across six generations, underscoring its genetic predisposition [3]. Similarly, a familial link to POM was observed in our study (104, 41.6%). Although the prevalence of familial consanguinity was only four (1.6%), its potential impact on genetic susceptibility should not be overlooked and must be investigated, as not many studies have included this as a risk factor. 

Occupation and the lifestyle of an individual also influence the development of POM, especially with jobs involving prolonged sun exposure or extended periods of screen time. Adequate sleep promotes mental restfulness and physical recovery including tissue repair and growth and skin rejuvenation. The average sleep duration observed was 6.35 hours. Insufficient duration of sleep can disrupt the circadian rhythm, leading to an increase in cortisol levels which may aggravate POM. Regularly engaging with motion pictures or texts increases the accommodation reflex, causing a strain on the periocular muscles. Frequent complaints of tiredness and eye fatigue were observed in the study due to the use of online study materials, television, and electronics for extended periods. Therefore, prolonged screen time contributes to the development and increased severity of POM. Bixonimania is an emerging form of POM linked to blue light exposure; further research on the mechanism is underway [4]. The regular eye rubbing habit has also been implicated in developing POM, possibly due to environmental factors or compulsive behavior.

Systemic diseases, autoimmune conditions, and vitamin deficiencies have often been linked to the development of POM. With 98 (39.2%) cases associated with systemic diseases, anemia was most prevalent, seen in 26 (10.4%) patients. POM may result from pallor which imparts a darker hue to the periocular area due to insufficient perfusion of oxygen in the periocular tissues [2]. An atopy diathesis was seen in eight (3.2%) patients which included atopic dermatitis, recurrent rhinitis, and asthma; on the contrary, 19 (19%) were reported by another study [5]. In Graves' disease, serum TSH is typically low, while adrenocorticotropic hormone levels are elevated, which increases the melanotropic activity causing POM; this is also known as the Jellinek sign [6]. With 22 (8.8%) patients with thyroid disorder, elevated serum TSH in two (0.8%) and decreased serum TSH in five (2%) were observed. During an acute infection, the body releases prostanoids, cytokines, chemokines, and other inflammatory mediators which in turn increases the melanocyte activity; reactive oxygen species are also generated during the inflammatory phase which may contribute to the development of POM post-infection.

An increase in the darkening of POM in the pre-menstrual period may occur due to vascular stasis and extravasation of blood, especially in the vascular type of POM [7]. Similarly, 71 (28.4%) patients reported worsening of POM during menstrual and pre-menstrual periods. Fewer studies have explored the association between menstruation and the type of POM, which can provide valuable insights into the underlying pathophysiology. Exposure to ultraviolet radiation increases the synthesis of corticotrophin, alpha-melanocyte-stimulating hormone, and interleukin-1, all of which may contribute to an increase in the formation of melanin, thereby worsening POM. The parameter used for significant sun exposure was 4-6 hours per day wherein 72 (28.8%) patients reported the same. Certain drugs, such as topical anti-glaucoma medications like latanoprost and bimatoprost, have been implicated in causing temporary POM. In addition to this, minocycline, antipsychotic drugs, chemotherapy drugs, prostaglandins, psoralens, oral contraceptives, and hormone replacement therapy are also known to contribute to POM. Forty-eight (19.2%) patients had a history of drug use for systemic diseases which included anti-hypertensives, oral hypoglycemic drugs, oral contraceptive pills (OCP), and antithyroid drugs. A study reported the development of POM in a patient after using OCP for six months [8]. Additionally, 94 (37.6%) patients used self-prescribed topical steroids (clobetasol propionate, fluocinonide, and combination preparations among others) and certain topicals that are falsely publicized to correct POM altogether, often purchased based on recommendations from others.

An anatomy-based physical examination of POM can be classified into four types, tear trough, shadow, visible lower eyelid bulge, and dermatochalasis, among which tear trough was the most prevalent (229, 91.6%). The site of involvement of POM is varied across studies and is also perceived differently based on the angle of lighting and skin laxity; therefore, emphasis on performing the manual stretch test in natural lighting must be made. POM is of four types, constitutional, post-inflammatory, vascular, and shadow, out of which the constitutional type of POM was the predominating type. While some studies frequently observed the post-inflammatory type of POM, Ranu et al. found the vascular type to be the most prevalent [9,10]. Grading of POM includes mild (mild lower eyelid pigmentation), moderate (pronounced pigmentation), severe (deep pigmentation involving all eyelids), and very severe (pigmentation extending beyond the infraorbital fold). The mild type was the most common POM grade observed (144, 57.6%) (Figure 1), in comparison to 40 (40%) and 22 (11%) cases in studies by Ramakrishnan et al. and Sheth et al., respectively [5,11]. Screen time showed a significant association with the severity of POM (p=0.004), with the severe grade of POM averaging 6.62±3.37 hours of screen time. Wood's lamp examination helped to differentiate between the epidermal and dermal types of pigmentation in POM, wherein 180 (72%) had the dermal type and 70 (28%) had the epidermal type of pigmentation (Figure 2 and Figure 3); however, a study reported 100 (100%) cases with the dermal type [8].

Dermoscopy is a non-invasive and reliable tool for the diagnosis of various dermatoses. One can demonstrate pigmentary patterns, vasculature, and skin surface markings and arrive at a diagnosis of various types of POM, which is known to be challenging by simply visualizing through the naked eye. Pigmentary patterns are commonly associated with the constitutional and post-inflammatory type of POM. At least 70% of patients had more than one type of pigmentary pattern with an increased frequency of blotches (166, 66.4%) and fine speckled (30, 12%). Similar observations were made by Jage and Mahajan, but with common findings of blotches and exaggerated pigment networks [9]. Among the vasculature patterns, telangiectasia and superficial dilated veins are frequently seen in the vascular type of POM. The prevalence of telangiectasia in the present study is relatively higher (211, 84.4%) as compared to the other studies [9], which may be attributed to the side effects of the application of home remedies (125, 50%) and topical medications (94, 37.6%). With a mean duration of 6.82 years, a correlation may exist between the prolonged use of topical medications and the observed changes. Exaggerated skin markings may be inflicted due to secondary actions of constant eye rubbing, history of atopy, and post-steroid abuse. However, no atrophic changes were observed despite a history of topical steroid use.

With POM drawing attention to the face, it can undermine patient confidence causing anxiety and stress, further affecting their societal relations and lowering their quality of life. The average MELASQoL score was found to be 25.63±10.52, categorized as the mild grade. A significant association was observed between the grade of POM and the MELASQoL scores, with higher grades of POM correlating with greater impairment in the quality of life (p<0.00). Most participants with grade 1 POM experienced mild impairment, whereas those with grade 3 POM showed moderate to severe impairment. However, not many studies have observed the effects on quality of life using the MELASQoL scale in patients with POM.

Stress is subjective and the perception of a certain grade of stress differs from person to person. PSS was developed by Sheldon Cohen, Tom Kamarck, and Robin Mermelstein in 1983 which assesses the impact of various circumstances on people's emotions and sense of stress. PSS in the study observed 114 (45.6%) patients with slightly higher-than-average stress, with a mean score of 16.64±3.28. This aligns with Sharma and Raina, where the mean score was 19.2 and 106 (71.3%) experienced higher-than-average stress, but did not show an association [12]. Conversely, the association between the POM grading and PSS scores in the present study was not significant (p>0.05), indicating that stress levels did not significantly differ across POM grades. This suggests that other factors may influence stress levels rather than the severity of POM alone and stress is subjective.

Patients with body dysmorphic disorder (BDD) generally exhibit recurrent obsessive actions in an attempt to conceal, improve, or examine the problem. Repeatedly checking one's reflection, comparing oneself to others, extensive grooming, and needing constant reassurance are typical instances of these habits. The prevalence of BDD in general dermatology clinics and outpatient departments is around 9-12% [13]. The study found a prevalence of BDD in four (1.6%) patients. However, no indexed articles were found that assessed BDD in POM patients. Its presence underscores the need for a comprehensive approach to patient care, addressing both the psychological and physical aspects of POM.

The study location was situated in a rural area and saw a predominance of rural residents. The diagnosis of POM was based on clinical parameters only which does not exclude the possibility of rare differentials like localized amyloid deposition which can only be excluded by histopathological examination. In addition to this, histopathological examination will help differentiate between different types of deposition (like hemosiderin and melanin) aiding in targeted management. Similarly, ultrasonography evaluation was not done which would have given more information on the anatomical variations in various types of POM including pre-septal thickening, prolapsed retro-septal fat pad, infraorbital palpebral bags, and edema in the periorbital area. Since this is a descriptive study, no control group was present which could have yielded precise results.

## Conclusions

POM is a common but poorly understood dermatological condition influenced by various demographic and clinical factors. The psychological impact and underlying mechanisms of POM are underexplored, which is depicted by the disparity between 150 million search engine results on dark circle treatments and only around 100 indexed articles for the same. POM is a chronic cosmetic dermatosis for which multimodal treatments are available, yet have ineffective outcomes. POM is not just a cosmetic concern but can also indicate underlying health issues that are often overlooked which warrants a thorough investigation. Patients often experience significant frustration with POM, impacting their daily activities, making it important to screen these individuals for BDD. With the diversity in the skin types among the Indian population and varied demography, further inclusive studies are needed to establish a definitive POM classification for more effective treatment.
